The article "A Study on the Personality Traits and Their Influencing Factors of Children from Poor Families from the Perspective of Psychological Education" was published in 2022. Journal: J Healthc Eng.

# A Study on the Personality Traits and Their Influencing Factors of Children from Poor Families from the Perspective of Psychological Education

**DOI:** 10.1155/2022/3002993

**Published:** 2022-01-25

**Authors:** Huiling Fan, Zhiyuan Xu

**Affiliations:** ^1^School of Marxism, Wuhan University of Technology, Wuhan 430000, China; ^2^“Research Center of Cultural Construction and Social Governance in Ethnic Areas” as the Key Research Base of Humanities and Social Sciences in Guangxi Universities, Guangxi, Nanning, China

## Abstract

The problem of poor children's psychological development has been widely concerned by governments all over the world. At present, the research results of poor children's psychological development show that poor children mainly have cognitive, mental health, and behavioral problems. This paper studies the personality traits and their influencing factors of children from poor families from the perspective of psychological education. By giving the definition of children from poor families and poor families, this paper analyzes the psychological development of poor children, analyzes the personality traits and influencing factors of children from poor families from the perspective of psychological education, obtains the standard scores of 16 personality traits and their dimensional personality factors and personality factors, and uses the clustering method to realize the difference analysis of personality characteristics of various samples. From the perspective of quantitative psychological education, this paper analyzes the correlation between personality traits and influencing factors of children from poor families in order to provide basis and reference for the government and society to implement targeted poverty alleviation and cut off the intergenerational transmission of poverty.

## 1. Introduction

“China's children's population in 2015 facts and data” points out: “in 2015, the number of permanent children living in poverty-stricken areas in China is roughly estimated to be 65 million, accounting for 24% of China's children population, of which 68% live in rural poverty-stricken areas. Considering that not all children living in poverty-stricken areas are poor, roughly 15 million children are in poverty, their survival and development status is particularly worthy of attention” [1]. Poverty is one of the biggest obstacles to children's survival and development. Young and vulnerable make children more vulnerable to the impact of poverty. Therefore, poor children suffer from not only material shortage but also lack of spirit and emotion, and the impact is irreversible.

Studies on the influencing factors of the early development of poor children mainly focus on the fields of sociology, neuroscience, public management, and psychology [2]. The social structure and interpersonal relationship caused by family poverty affect children's physical and brain development through repeated pressure, which leads to social replication or intergenerational transmission of poverty, so that parents' social class can predict children's social class. Rinaldi et al. [3] believe that the problem of poor children has become a hot and important issue in the new era. It is of theoretical and practical significance to study the influencing factors of poor children's psychological development. Analyzing the psychological development of poor children from the perspective of psychological theory is helpful to solve the misunderstanding about poor children. In practice, the “lost childhood” of poor children is the pain of the family and the difficulty of national development [4]. It is also an important link for the party and the government to pay attention to early poverty and implement early poverty alleviation in order to cut off the vicious circle of “poverty growth retardation lifelong poverty intergenerational transmission” and achieve and consolidate the goal of comprehensively getting rid of poverty.

To this end, this paper reviews the relevant research at home and abroad, summarizes the influencing factors of poor children's psychological development, and tries to put forward the countermeasures of eliminating poverty on children's psychological development and the new direction of future research in order to provide the basis and reference for the government and society to implement targeted poverty alleviation, help the poor first, and block the intergenerational transmission of poverty and other practical activities.

## 2. The Definition of Poor Children and the Analysis of Their Psychological Development

### 2.1. Definition of Poverty

The phenomenon of “poverty” has always been the focus of political economics, economics, sociology, and other disciplines. Especially at present, China is in the period of social transformation. Special groups produced with economic poverty, such as poor primary school students, left-behind children, and urban migrant children, have attracted the general attention of all sectors of society. With the deepening of research, the understanding of poverty is becoming more and more profound. The definition of “poverty” has expanded from a single lack of material objects and income to a lack of capacity, but a more consistent view of the concept of “poverty” has not been formed. This is mainly due to the historical and relative characteristics of the concept of poverty. The so-called historicity means that the judgment of poverty is influenced by the national conditions, cultural background, and the development level of productive forces, showing the characteristics of stages; and relativity means that poverty is relative to individuals or groups in the same environment. Due to different levels of productivity development, different social groups have different degrees of satisfaction with their living needs, thus showing the gap between the rich and the poor [5, 6]. Therefore, there are obvious differences between different disciplines in the interpretation of poverty. From the existing research literature, the research on the phenomenon of “poverty” and the criteria for identifying whether it is “poverty” are mainly from the perspective of economics [7–9]. Generally speaking, poverty means that the living conditions that an individual or family can achieve are lower than the socially acceptable living standards.

### 2.2. The Concept of Poor Children

Because there are absolute and relative poverty standards, especially there are still great differences in poverty status and actual standards between urban and rural areas and regions, it is not easy to identify a scientific and unified concept of poor children. Based on the research subject and the actual situation of children in distress, this paper nodes poor children as all children whose family income is lower than the local minimum living security standard.

From the perspective of physical and psychological development and maturity, children are a special group. Their growth is affected by family environment and early experience, among which family poverty and poor experience are important factors threatening their physical and mental health and development. The lack of conceptualization and debate on the particularity of children's poverty has had a great impact on China's poverty alleviation policies. At the same time, the success of China's poverty alleviation policies has partially hindered the comprehensive understanding of children and families, which leads to the fragmentary understanding of the connotation and nature of poverty, that is, taking family income as an important measure. However, with the deepening of poverty research, people realize that it is far from enough to measure children's poverty simply by the single dimension of family socioeconomic status or family income. Moreover, children may not necessarily get their due share of family income and benefit from it. The concept of adult poverty and child poverty may be confused [10–15]. Therefore, the understanding and definition of poor children has become an important issue in this field, and a scientific definition of poor children is of great significance for the government to formulate policies aimed at improving children's well-being.

There are two views on the concept of poor children. The first is to measure children's poverty based on monetary method. The monetary method is the most common method to determine and measure poverty at national and international level. In practice, poor children are defined as all children whose family income is lower than the local minimum living standard according to their family income, mainly including children in urban and rural families, left-behind children in rural areas, orphans, and children affected by AIDS [16, 17]. However, poverty is a comprehensive phenomenon of social material life and spiritual life. It is easy to ignore the gender, family structure, age, and other factors of poor children only by the monetary method. The second is to measure children's poverty based on the method of rights deprivation, that is, to integrate the concept, analysis, values, and language of human rights into poverty reduction and poverty alleviation dialogue, which is essentially a poverty alleviation method based on human rights. The United Nations Children's Fund uses a “Bristol index” as a method to measure deprivation of rights and puts forward eight indicators, including food, education, safe drinking water, sanitation, health care, housing, information, and access to services, as an important basis to judge whether children are absolutely poor [18]. This view expands the one-dimensional concept of poor children based on family income.

### 2.3. Psychological Development of Poor Children

As a special group, poor children's poverty experience or situation has a negative impact on their physical and mental health. Duncan and Brooks Gunn (1997) are the first scholars to extensively study the possible long-term consequences of early childhood poverty. Duncan et al. (2010) conducted a longitudinal dynamic group study on children living in poverty from birth to 5 years old. The correlation between family income and children's achievement in early childhood is higher than that between family income and mental health [19–22]. Johnson et al. (2016) also found that poor children are more likely to experience worse health conditions, more severe developmental delay, lower achievement, and more behavioral and emotional problems than normal children [23, 24]. Since then, a large number of literatures have revealed the relationship between early poverty and mental health, cognitive development effect from the aspects of mental health, and brain development of poor children.

## 3. Influence of Psychological Education on the Personality Traits and Influencing Factors of Children from Poor Families

Due to the specific environment in which poor children live and their own psychological characteristics, their mental health is far lower than that of ordinary children. Generally, poor children do not have enough confidence and belief in life and future. They always think that they are marginal members of society and are difficult to integrate into the whole society. Among the poor children, they can better complete the nine-year compulsory education, but few can really enter high school and university. They do not have the basic conditions and competitiveness in the fierce employment competition. This is because it is difficult for poor children to feel the real warmth of their family when they grow up, and they often have problems such as withdrawn personality and psychological closure. When most poor children get along with others, they get sympathy and compassion, but at the same time they do not get the minimum respect and equality, so it is difficult to integrate into the society.

There is no doubt that the survival and development of poor children are affected by various aspects and the internal mechanism of the negative impact is of more research value [25]. Previous studies mainly explained this problem from the perspectives of family and environmental pressure, family education and investment, and poverty culture social factors are analyzed, and some solutions are given.

1. *Personal factors*. In the observation and interview of poor children, it is found that most of the formation of inferiority comes from children's unreasonable beliefs about themselves. In the interview, the author found that children will attribute a series of bad things around them to themselves, resulting in self-denial and negative emotions. Under the guidance of ABC personality theory, we will help poor children eliminate their inferiority complex and enhance their self-confidence through rational treatment.
2. *Family factors*. Increase financial support for families with special children, especially for low-income families and poor families. In ethnic areas, families with special children have relatively less financial resources, which has become the main source of parents' psychological pressure, and a good and stable economic foundation is also the main pillar of education and rehabilitation training for special children. Therefore, the government's financial support is one of the important ways to relieve the psychological pressure of parents of special children. According to Grendel's family stress model, low economic status constitutes stress experience, and sense of control and powerlessness are the core functions of vulnerability of low-status people. Poor children are more likely to live in more chaotic, structural, and crowded families than their peers. The instability of family structure and poor school environment due to economic deficiency cause repeated pressure on poor children, and pressure promotes adaptation. However, poverty and its long-term chronic pressure will cause frequent or continuous activation of biological stress system. The damage of biological stress response system function is considered to be a central mechanism of human development affected by exposure to adverse early living environment. Long-term stress will lead to body wear, affecting the development of the nervous system and brain.
3. *Community factors*. The community and competent departments can regularly guide parents of special children to participate in parent mutual aid group activities, help each other through emotional exchange, and experience discussion, so that parents can experience higher subjectivity, so as to bring this positive and optimistic attitude to children's education and rehabilitation training.
4. *School factors*. School is an important place for children to learn and grow up, where children will learn knowledge and rules and constantly complete their socialization. Therefore, the guiding role of school for children is very important. In comparison, poor children will have inferiority complex and gradually do not recognize and deny themselves. Therefore, we need to strengthen the publicity and popularization of psychological knowledge in schools, help children establish a correct world outlook, values and outlook on life, help children sort out their emotions in time, change their misconceptions, and guide them to identify with themselves, affirm themselves, and believe in themselves.
5. *Social factors*. Social support system is a huge and complex system, which is based on the resources owned by individuals. At the same time, it also has an impact on individual life, learning, communication, and other aspects. Improve the social service security system, and improve the laws and regulations related to special children. The laws and regulations of government departments can more specifically and operationally regulate the rights of special children and their families and effectively safeguard and protect these rights and interests, so as to reduce the psychological pressure of parents of special children, especially the parents of poor special children.

## 4. Empirical Analysis

### 4.1. Research Object and Experimental Parameters

The college conducted a random survey of poor children in school. At the same time, attention should be paid to balance the distribution of subjects in gender, grade, subject, and source of students. The survey lasted for nearly one month from early May 2020 to early June 2021. In this paper, through group testing and random sampling, 2000 questionnaires were distributed, 1600 questionnaires were returned, and 1584 questionnaires were valid, with an effective questionnaire rate of 92.53%. The subjects came from different majors. The distribution of the subjects in the variables of gender, grade, subject, and place of origin is shown in Table 1.

The above data are used for the next experimental verification.

### 4.2. Data Processing

The above experimental data are stored in the SQL database of Excel. SPSS 20.0 online data analysis is used to analyze the above experimental data. Descriptive statistics, *z* test, correlation analysis, confirmatory factor analysis, and other statistical methods are used to study the personality traits of poor children. The average standard score of children from poor families is shown in Table 2.

It can be seen from Table 2 that the standard scores of 16 personality traits of children from poor families are between 3.5632 and 5.542. The standard scores of the four dimensional personality factor types ranged from 3.2421 to 7.5421, indicating that the poor primary school students were also at the middle level in 16 personality traits and four dimensional personality factor types. Among the four personality factors, the score of personality factors of mental health was slightly higher than the average score of 26 points. The scores of professional achievers and those who have the ability to grow in the new environment are lower than the corresponding average scores of 62 and 31. The score of personality factors of the creative strong is 7 after the conversion, which indicates the mental health of poor primary school students.

The study conducted cluster analysis on 16 personality traits and their dimensional personality factors and personality factors to describe the main types of personality characteristics of poor primary school students.

Firstly, 150 samples are selected by the random number table method, and the classification number is preliminarily determined by the hierarchical clustering method. The results show that it is feasible to divide the samples into 3 categories, 4 categories, and 5 categories. Then, according to category 3 the results show that it is reasonable to divide the samples into three categories, and the difference of personality traits between each type reaches a significant level (*P* < 001); at the same time, the number of poor primary school students of all types is roughly the same. After clustering, descriptive statistics and F-tests are carried out on the personality traits, dimensional personality factors, and personality factors of various samples. The results are shown in Table 3.

In order to further explore the degree of difference between various types of personality characteristics of poor primary school students, the data are tested afterwards. It can be seen from Tables 2 and 3 that the scores of these three personality types on 16 personality traits and their dimensional personality factors are almost statistically significant (*P* < 0.05 − 0.001). In addition, we also use the results of category analysis to verify the reliability of the classification number “3”. The results show that it is the best choice to divide the personality traits of poor primary school students into three categories.

## 5. Conclusion

From the above experimental results, we can see that from the perspective of psychological education, there are five main factors affecting the personality traits of children from poor families, including personal factors, family factors, community factors, school factors, and social factors. Among them, personal factors are the most important, while family factors and school factors also occupy a certain proportion. It shows that poor children's inner thoughts and external environment have an important impact on their growth, and it plays an important role in improving the external environment for children from poor families.

## Figures and Tables

**Table 1:** Basic information of subjects.

Project	Variable	Number of people	Proportion
Gender	Male	786	49.62%
	Female	798	49.81%
Grade	1	297	18.75%
	2	210	13.26%
	3	220	13.89%
	4	210	13.26%
	5	259	16.35%
	6	388	24.50%
Subject	Mathematics	432	27.27%
	Grammar	653	42.22%
	English	499	31.50%
Source of students	Town	321	20/27%
	Countryside	1261	79.61%
	Not filled in	2	1.26%

**Table 2:** The standard scores of 16 personality traits, dimensional personality factors, and personality factors of poor children.

Personality factors	Number of valid copies	Minimum value	Maximum	Average value
Music group	1584	2.00	15.00	5.584
Intelligence	1584	2.00	12.00	5.462
Stability	1584	2.00	14.00	5.763
Bullying	1584	2.00	12.00	5.436
Excitability	1584	2.00	8.00	6.324
There is constancy	1584	2.00	15.00	6.321
Daring	1584	2.00	15.00	5.175
Susceptibility	1584	2.00	15.00	7.133
Skepticism	1584	2.00	8.00	8.521
Fantasy	1584	2.00	8.00	5.326
Privateness	1584	2.00	8.00	5.175
Anxiety	1584	2.00	15.00	7.421
Experimental	1584	2.00	15.00	8.421
Independence	1584	2.00	15.00	5.557
Self-discipline	1584	2.00	15.00	5.325
Tensity	1584	2.00	15.00	5.432
Adaptation and anxiety	1584	0.43	68.12	1.453
Introversion and extroversion	1584	0.65	87.99	1.543
Sentimental and serene alert	1584	0.63	6.55	4.453
Cowardly and decisive	1584	0.53	6.88	55.321
Personality factors of mental health people	1584	5.32	7.39	55.432
Personality factors of professional and accomplished persons	1584	16.43	6.88	51.432
Personality factors of the creative strong	1584	58.55	76.00	76.675
Ability to grow in a new environment	1584	68.00	78.43	22.433
The personality factors of the students				

**Table 3:** Analysis on the differences of personality characteristics of different samples after clustering.

Personality factors	Type I (*n* = 558)	Type II (*n* = 579)	Type III (*n* = 536)	F Value
Music group	6.21 ± 1.22	6.31 ± 1.65	6.32 ± 1.44	135.343*∗∗∗*
Intelligence	5.58 ± 1.21	5.23 ± 1.11	4.25 ± 1.32	187.654*∗∗∗*
Stability	3.38 ± 1.02	5.43 ± 1.65	5.65 ± 1.76	423.214*∗∗∗*
Bullying	3.93 ± 1.53	4.87 ± 1.43	6.21 ± 1.66	29.762*∗∗∗*
Excitability	4.22 ± 1.89	3.86 ± 1.54	5.12 ± 1.43	189.432*∗∗∗*
There is constancy	4.62 ± 1.65	4.66 ± 1.65	5.76 ± 1.54	267.875*∗∗∗*
Daring	3.86 ± 1.22	5.33 ± 1.62	6.12 ± 1.78	156.887*∗∗∗*
Susceptibility	5.65 ± 1.99	5.76 ± 1.76	7.21 ± 1.99	108.432*∗∗∗*
Skepticism	5.43 ± 1.73	4.32 ± 1.72	6.11 ± 1.88	63.211*∗∗∗*
Fantasy	5.66 ± 1.32	5.21 ± 1.62	3.21 ± 1.46	33.632*∗∗∗*
Privateness	4.33 ± 1.32	4.77 ± 1.43	5.44 ± 1.64	25.541*∗∗∗*
Anxiety	3.28 ± 1.53	4.56 ± 1.23	5.21 ± 1.43	264.234*∗∗∗*
Experimental	5.66 ± 1.22	3.65 ± 1.64	6.31 ± 1.66	41.321
Independence	6.08 ± 1.54	2.88 ± 1.32	5.21 ± 1.97	324.542*∗∗∗*
Self-discipline	4.55 ± 1.64	3.65 ± 1.76	5.22 ± 1.54	307.212*∗∗∗*
Tensity	3.77 ± 1.54	4.21 ± 1.72	5.12 ± 1.32	575.432*∗∗∗*
Adaptation and anxiety	4.66 ± 1.32	8.33 ± 1.43	6.21 ± 1.43	465.334*∗∗∗*
Introversion and extroversion	5.43 ± 1.34	7.41 ± 1.23	8.42 ± 1.54	286.321*∗∗∗*
Sentimental and serene alert	6.33 ± 1.65	6.44 ± 1.53	8.21 ± 1.76	431.765*∗∗∗*
Cowardly and decisive	4.55 ± 1.32	5.34 ± 1.12	4.87 ± 1.66	546.321*∗∗∗*
Personality of mental health people	5.32 ± 1.65	5.23 ± 1.23	6.87 ± 3.87	121.534*∗∗∗*
The specialty has the personality of an achiever	3.97 ± 1.99	6.76 ± 1.43	5.87 ± 1.66	234.642*∗∗∗*
The personality of the creative strong	5.11 ± 1.65	4.32 ± 1.53	6.84 ± 1.21	421.453*∗∗∗*
Ability to grow in new environment	11.87 ± 1.55	4.23 ± 1.21	5.14 ± 1.76	278.643*∗∗∗*
Class size	32.542%	30.241%	37.217	-

*∗P* < 0.05, *∗∗P* < 0.01, and *∗∗P* < 0.001; in the LSD test, “1” represents type I, “2” represents type II, and “3” represents type III.

## Data Availability

The data sets used and analyzed during the current study are available from the corresponding author on reasonable request.
